This article has been retracted.

# Functional Analysis of Bronchopulmonary Dysplasia-Related Neuropeptides in Preterm Infants and miRNA-Based Diagnostic Model Construction

**DOI:** 10.1155/2022/5682599

**Published:** 2022-04-25

**Authors:** Yue Zhang, Xiangyong Kong, Jie Zhang, Xu Wang

**Affiliations:** ^1^Department of Neonatal Intensive Care Unit, Beijing Aiyuhua Maternal and Children Hospital, Beijing, China; ^2^BaYi Children's Hospital, Seventh Medical Center of Chinese PLA General Hospital, China

## Abstract

**Background:**

Bronchopulmonary dysplasia (BPD) has a high mortality rate. This study was aimed at identifying and analysing the risk factors associated with BPD using bioinformatic and mechanical analyses and establishing a predictive model to assess the risk of BPD in preterm infants.

**Methods:**

We identified differentially expressed RNAs via the intersection of miRNAs between datasets. Online analysis tools were used to predict genes targeted by differentially expressed miRNAs (DEmiRNAs) and to generate and visualise competing endogenous RNA (ceRNA) coexpression networks. Gene Ontology (GO) and Kyoto Encyclopedia of Genes and Genomes (KEGG) analyses were subsequently performed on the DEmiRNAs. In addition, an intersection analysis was performed on mRNA and neuropeptide-related genes in the ceRNA network. DEmiRNAs associated with BPD and those involved in ceRNA networks were used to establish a diagnostic prediction model. The GSE108604 dataset was used as a validation set to verify the model.

**Results:**

A total of 26 DEmiRNAs were identified from the tracheal aspirates (TAs) of patients with BPD and healthy controls. In addition, a total of 1076 DEmRNAs were obtained from the GSE8586 dataset. Functional enrichment analysis of DEmRNAs revealed an abnormal reduction in mitochondrial-related activity and cellular responses to oxidative stress in patients with BPD. The neuropeptide-related genes *OPRL1* and *NPPA* were found to be upregulated in BPD samples. Eventually, hsa-miR-1258, hsa-miR-298, hsa-miR-483-3p, and hsa-miR-769-5p were screened out and used to establish the prediction model. Calibration curves and detrended correspondence analysis (DCA) revealed that the model had good clinical applicability.

**Conclusions:**

The prediction model provided a simple method for individualised assessment, early diagnosis, and prevention of BPD risk in preterm infants.

## 1. Introduction

Bronchopulmonary dysplasia (BPD) is a chronic lung disease that is one of the most common and adverse consequences of preterm birth. Owing to the widespread use of mechanical ventilation in the neonatal intensive care unit (NICU) and the increased survival rate of infants with very low birth weight (VLBW), the incidence of BPD has increased. BPD is diagnosed in almost 80% of preterm infants that are born between 22 and 24 weeks of gestation [1]. BPD has a high mortality rate, and patients who survive are more likely to develop extrauterine growth retardation and have a significantly higher risk of developing respiratory and neurological abnormalities, which adversely affects the quality of life of the child [2]. Therefore, early identification of preterm infants having a risk of BPD and adopting proactive measures are essential for improving the prognosis. Moreover, reducing the incidence of BPD is one of the major challenges in the NICU.

Although the pathogenesis of BPD remains unclear, the expression of various neuropeptides was found to be abnormal during the development of BPD [3–6]. Many studies based on traditional research methods have found that neuropeptides can be used as potential biomarkers for BPD [6–8]. In addition to the traditional approaches, large data-based bioinformatic mining has been developed rapidly in the past decades and has promised to overcome the existing barriers. A neural network is one of the many machine-learning algorithms that can be used for both supervised and unsupervised tasks such as classification and visual recognition and can handle complex nonlinear problems [9]. Machine-learning models can naturally handle the richness and complexity of digitalised patient data by learning predictive patterns in the data, which in turn can be used to build individualised prediction models [10–12]. We suggest that neuropeptides, as biomarkers of BPD, may be a comprehensive predictor of BPD prognosis. The Gene Expression Omnibus (GEO) database contains microarray, massive parallel sequencing (MPS), and other high-throughput sequencing data which was used in this study.

This study is aimed at identifying the risk factors associated with BPD using a bioinformatic approach and establishing a predictive model for individualised assessment of the risk of BPD and its early prevention in preterm infants.

## 2. Methods

### 2.1. Patient Information and Data Preprocessing

All datasets related to BPD in the GEO database were considered for inclusion in this study. The RNA profile data and clinical information of patients with BPD were downloaded from GEO (https://www.ncbi.nlm.nih.gov/geo/). The exclusion criteria were as follows: (a) patients with no presumed clinical diagnosis, (b) patients with critical illnesses other than BPD, and (c) patients with incomplete RNA data, including transcriptional data of miRNA and mRNA. miRNAs that were coexpressed among the datasets, including GSE156055 [13], GSE165828 [14], and GSE108604 [15], were identified and subsequently analysed. The GSE156055 dataset includes miRNA profiles in tracheal aspirates (TAs) from 51 infants who underwent invasive mechanical ventilation. Among these, 25 preterm infants were diagnosed with BPD and 26 full-term infants received invasive mechanical ventilation for elective surgery. The GSE165828 dataset includes miRNA profiles in tracheal inhalations (TAs) from 25 very preterm infants receiving invasive mechanical ventilation. Eight of these infants were diagnosed with mild/moderate BPD, and 17 were diagnosed with severe BPD. The GSE108604 dataset is based on a prospective cohort study, which performed miRNA profiling on approximately 800 miRNAs from 18 samples (including 9 patients with BPD). The GSE8586 dataset includes 54 cases of umbilical cord tissue (20 of which are BPD patients). GSE156055 and GSE165828 were used as test sets for variance analysis and model construction. GSE108604 was used as a validation set to validate various machine-learning models. In addition, the mRNA-seq data were downloaded from the GSE8586 dataset and used for mRNA-related analyses [16].

### 2.2. Identification of Differentially Expressed RNAs

Differentially expressed miRNAs (DEmiRNAs) between the BPD and control groups were analysed using the “edgeR” and “limma” packages in R software. Platform annotation files corresponding to the transcriptional data were used to define and annotate miRNAs and mRNAs through a program code written in the Perl software. Differences in the expression of these miRNAs and mRNAs were defined as significant based on fold change (FC) and associated *P* values. In the preliminary screening, statistical significance was set at *P* < 0.05. The DERNA expression profiles were normalised and batch corrected via log transformation. The “heat map” and “gplots” functions of the R package were used to generate volcano maps of DEmiRNAs.

### 2.3. Filtering of Neuropeptide Gene Sets

To screen for a wide range of neuropeptide-related genes, we conducted a literature review and Wikipedia (https://en.wikipedia.org/wiki/Neuropeptide) search. Through the literature review, we analysed previous studies on neuropeptides and included neuropeptides that may be related to BPD in the gene set. The main neuropeptides we considered were opioid peptides, kinins, neuropeptide Y (NPY), substance P (SP), calcitonin-gene-related peptide (CGRP), atrial natriuretic peptide (ANP), brain natriuretic peptide (BNP), C-type natriuretic peptide (CNP), and their receptor genes [17–19].

### 2.4. Construction of ceRNA Network

Using online tools and databases such as miRWalk (http://mirwalk.umm.uni-heidelberg.de/), miRDB (http://www.mirdb.org/), miRTarBase (https://mirtarbase.cuhk.edu.cn/), and TargetScan (http://www.targetscan.org/), we predicted genes targeted by the identified DEmiRNAs. All predicted target genes were considered for further analysis to examine their possible mechanisms of action. The Cytoscape v3.6.0 software was used to generate and visualise competing endogenous RNA (ceRNA) coexpression networks [20].

### 2.5. Functional Analysis

To further elucidate the biological functions of coexpressed ceRNAs, we performed Gene Ontology (GO) enrichment and Kyoto Encyclopedia of Genes and Genomes (KEGG) pathway analyses. We used the R package “clusterProfiler” to perform Gene Set Enrichment Analysis (GSEA) on the target genes. The reference gene set curated for pathway annotation was c2.cp.v7.2.symbols.GMT. *P* < 0.05 was set as the cut-off criterion for defining significance.

### 2.6. Construction of a Diagnostic Prediction Model

DEmiRNAs associated with BPD and those involved in the ceRNA network were used to establish a diagnostic prediction model. Along with the R language software, several machine-learning models were used to predict diagnosis, including support vector machine recursive feature elimination (SVM-RFE), lasso regression, and logistic regression analysis as previous researches [21–23]. We used the SVM-RFE model to evaluate the number of diagnosis-related DEmiRNAs and subsequently analysed their predictive power based on the area under the curve (AUC) values. Lasso regression prevented overfitting by penalising the features incorporated into the model. In addition, univariate logistic regression models were used to determine the prognostic characteristics of DEmiRNAs. Those with *P* < 0.05 were considered as candidate variables and were included in the stepwise multivariate logistic regression analysis. miRNAs targeting nucleoprotein (NP) with *P* < 0.2 were included in the multivariate regression analysis. In addition, the odds ratio (OR) and 95% confidence interval (CI) of each DEmiRNA were evaluated. The performance of the three diagnostic prediction models, namely, SVM-RFE, lasso regression, and logistic regression analysis, was evaluated, and the best model was selected for subsequent analyses. A comprehensive prognostic scoring system (risk score) was established based on the DEmiRNAs of the optimal model. The risk score was calculated as follows: RiskScores = *β*_0_ + exp_miRNA1_ × *β*_miRNA1_ + exp_miRNA2_ × *β*_miRNA2_ + , ⋯exp_miRNAn_ × *β*_miRNAn_, where exp is the expression level and *β* is the regression coefficient derived from the multivariate logistic regression model. Receiver operating characteristic (ROC) curves were used to assess the sensitivity and specificity of miRNA signatures in BPD.

### 2.7. Validation of the Diagnostic Prediction Model

The GSE108604 dataset was used as a validation set to verify the predictive ability of the diagnostic model. Using the diagnostic prediction model obtained via analysis of the training set, samples in the validation set were distinguished between BPD and control samples. Subsequently, ROC curves were plotted for the entire cohort and training and validation sets to analyse the predictive power of the prediction models. The AUC values were used to compare the diagnostic classification ability among machine learning models.

### 2.8. Construction of a Nomogram

The parameters of the model with the best predictive power were selected, and a nomogram was generated using the “rms” package of the R software. A calibration curve was plotted to evaluate the predictive consistency of the nomogram. Eventually, DCA curves were plotted to assess the clinical utility and safety of the model [24].

### 2.9. Statistical Analysis

Differences in miRNA expression between the two groups were compared via one-way analysis of variance (ANOVA). Pearson correlation analysis was used to investigate the relationship among miRNAs in the ceRNA networks. Statistical analyses were performed using the R software version 4.0.5 (https://www.r-project.org/). We used the “pROC” software package to plot ROC curves for analysing the diagnostic performance of candidate DEmiRNAs. All tests performed for validating the hypothesis were two-sided, and *P* < 0.05 was considered statistically significant unless stated otherwise.

## 3. Results

### 3.1. Identification of BPD-Related DERNAs

A total of 94 tracheal aspirate (TA) samples were included from the GSE156055, GSE165828, and GSE108604 datasets, including 59 TA samples of preterm infants with BPD and 35 TA samples of healthy controls, for miRNA analysis. In addition, we obtained RNA-sequencing (RNA-seq) data of 54 umbilical cords of newborns with extremely small gestational age (20 with BPD and 30 without BPD) from the GSE8586 dataset for mRNA analysis. The workflow and overall study design are demonstrated in Figure 1. A total of 26 DEmiRNAs, including 15 upregulated and 11 downregulated miRNAs, were identified from the TA samples of patients with BPD and controls according to the cut-off threshold. The volcano map demonstrated the FC and *P* values of DEmiRNAs (Figure 2(a)). In addition, a total of 1076 DEmRNAs (457 upregulated and 619 downregulated mRNAs) were procured from the GSE8586 dataset, and the results are demonstrated in Figure 2(b). The heat map demonstrated the expression of miRNAs and mRNAs in BPD and control samples (Figures 2(c) and 2(d)). To understand the molecular mechanisms involved in BPD development, we further performed GO and KEGG pathway enrichment analyses on DEmRNAs. The results revealed that serine-type peptidase activity, serine-type endopeptidase activity, protein tyrosine kinase activity, ephrin receptor activity, and transmembrane ephrin receptor activity were upregulated in BPD. In addition, mitogen-activated protein (MAP) kinase phosphatase activity, mitochondrial inner membrane, response to reactive oxygen species, positive regulation of apoptotic signalling pathways, and cellular response to oxidative stress were downregulated in BPD (Figures 3(a) and 3(b)). We found an abnormal reduction in mitochondrial-related activity and cellular response to oxidative stress in patients with BPD.

### 3.2. miRNA-mRNA ceRNA Network

To examine the interaction between DEmiRNAs and DEmRNAs, we constructed a ceRNA network. We predicted the target mRNAs of the 26 DEmiRNAs using miRWalk, miRcode, miRDB, and miRTarBase. Possible interactions among these predicted mRNAs and the 1625 DEmRNAs were cross-verified, and the results revealed that 26 miRNAs and 517 DEmRNAs were involved in the ceRNA network. The correlation between the expression of these 26 DEmiRNAs is demonstrated in a heat map (Figure 3(c)). After miRNAs and mRNAs were identified according to ∣log_2_FC | >1 and >0.6, respectively, the Cytoscape software was used to visualise the relationship between the 23 DEmiRNAs and the 119 DEmRNAs in the ceRNA network (Figure 4(a)). The ceRNA network indicated possible interactions among DEmiRNAs in BPD. The upregulated and downregulated pathways in the network are demonstrated in Figures 4(b) and 4(c). Transmembrane ephrin receptor activity, transmembrane receptor protein tyrosine kinase activity, and pyruvate metabolism were upregulated in the ceRNA network. However, regulation of respiratory gaseous exchange, beta-catenin destruction complex, glucocorticoid receptor binding, and beta-catenin binding were downregulated in the ceRNA network. In addition, the expression of complex molecules associated with gas exchange was abnormally downregulated in the ceRNA network, whereas alanine metabolism was upregulated.

### 3.3. Neuropeptides in the ceRNA Network

We performed an intersection analysis on mRNAs and neuropeptide-related genes in the ceRNA network and extracted overlapping mRNAs and their corresponding miRNAs (Figure 5(a)). To investigate the function of NP in the ceRNA network, the expression of the neuropeptide-related genes *OPRL1* and *NPPA* was analysed in BPD and control samples. The results revealed that *OPRL1* and *NPPA* were upregulated in BPD samples (*P* < 0.05; Figure 5(b)). In addition, the AUC values of *OPRL1* and *NPPA* for the diagnostic efficacy of BPD were 0.666 and 0.663, respectively (Figure 5(c)). This finding suggested that *OPRL1* and *NPPA* predicted BPD to a certain extent. To further investigate the significance of *OPRL1* and *NPPA* in BPD progression, GSEA was performed to evaluate the expression of neuropeptide-related pathways. The results revealed that KEGG CYTOKINE CYTOKINE RECEPTOR INTERACTION and NABA ECM REGULATORS were downregulated in the group with increased *OPRL1* expression (Figure 5(d)), and KEGG NEUROACTIVE LIGAND RECEPTOR INTERACTION and REACTOME ADORA2B MEDIATED ANTI INFLAMMATORY CYTOKINES PRODUCTION were downregulated in the group with elevated *NPPA* expression (Figure 5(d)). These results indicated that the NPs in the ceRNA network were related to cytokine activity and immune response function.

### 3.4. Construction and Validation of the Predictive Model for the Diagnosis of BPD

To identify predictive markers with potential diagnostic value, we used machine learning models to assess the 26 miRNAs in the ceRNA network. The line graph representing the number of incorporated variables and the accuracy of the corresponding model during the training of the SVM-RFE model is demonstrated in Figure 6(a) (Table 1). The highest accuracy for diagnostic classification was achieved when 11 variables were included in the SVM model. The AUC value of the SVM model was 0.84 based on 11 variables for predicting the occurrence of BPD in the validation dataset. Similarly, lasso regression was used to penalise the variables to prevent overfitting (Figures 6(b) and 6(c)). Through lasso, principal component analysis (PCA) visualises the ability of SVM-RFE and the variables screened in distinguishing between patients with BPD and healthy individuals (Figures 6(d) and 6(e)).

We further performed univariate and multivariate logistic regression analyses to analyse the relationship between miRNAs and their diagnostic performance, and the results are demonstrated in Table 2. The NP-targeted miRNAs hsa-miR-650 (*P* = 0.088) and hsa-miR-769-5p (*P* = 0.156), with a cut-off value of *P* < 0.2 in the univariate analysis, were included in the multivariate analysis. Based on multivariate analysis, four variables were identified and included in the next step of logistic model construction. Among the 26 DEmiRNAs, four miRNAs, namely, hsa-miR-1258, hsa-miR-298, hsa-miR-483-3p, and hsa-miR-769-5p (Figure 7(a)), were eventually used to construct the miRNA-based diagnostic prediction model. The contribution of each of these four miRNAs in the diagnostic classification was demonstrated by ROC curves, and the corresponding AUC values were also calculated (Figure 7(b)). ROC curves were plotted to analyse the classification ability of the model. The diagnostic AUC of the four miRNA-based models in the entire cohort was 0.854 (Figure 7(c)). The AUC values of these four miRNAs that were combined for prediction were 0.850, 0.854, and 0.877 in the training, entire, and validation datasets, respectively. This finding revealed that the four miRNA models based on risk scores had good diagnostic predictive value (Figure 7(c)). Lastly, PCA was used to visualise their predictive ability in disease classification (Figure 7(d)).

### 3.5. Construction and Validation of a Nomogram

Based on previous analyses, we constructed a nomogram based on four miRNAs to predict the risk of BPD in preterm infants. In the model, hsa-miR-769-5p was the *NPPA*-targeted miRNA. Using the nomogram as a simple tool, we can better predict the occurrence and clinical management of BPD (Figure 8(a)). To analyse the accuracy and reliability of the nomogram as a clinical tool, we further used calibration curves and DCA for validation and evaluation. The calibration curve demonstrated an agreement between the predicted and observed results of the model for BPD diagnosis (Figure 8(b)). DCA revealed that the model had good clinical applicability (Figure 8(c)). These results implied that the constructed model can be used to predict the probability, diagnosis, and intervention of BPD in newborns as early as possible. In addition, the prediction model established using miRNAs provided new ideas and directions for further investigation on the underlying mechanisms of BPD development.

## 4. Discussion

Children with BPD have a higher prevalence of neurological deficits (motor, visual, and hearing dysfunction) and lower IQ scores and are more likely to develop learning difficulties and articulation delay [25–29]. The occurrence of BPD is a long-term and devastating burden on the family and society. Therefore, early identification of patients having a high risk of BPD and implementation of preventive measures are particularly significant. The Score for Neonatal Acute Physiology and Perinatal Extension II (SNAPPE-II) is an advanced neonatal scoring system used worldwide; however, it lacks specificity for BPD. This study developed a BPD risk prediction tool based on database and bioinformatic analyses for early diagnosis and individualised treatment of BPD.

In this study, hsa-miR-1258, hsa-miR-298, hsa-miR-483-3p, and hsa-miR-769-5p were selected, and a miRNA-based diagnostic prediction model with good diagnostic predictive value was constructed. In addition, neuropeptides related to *OPRL1* and *NPPA* were upregulated in BPD samples, and hsa-miR-769-5p was the *NPPA*-targeted miRNA in the model.

Neuropeptides have been found to play an important role in the pathological process of BPD. We speculate that the translation process of neuropeptides may be regulated by miRNAs. hsa-miR-630, hsa-miR-650, and hsa-miR-769-5p were found to be differentially expressed in BPD patients. In the present study, hsa-miR-650 and hsa-miR-630 were found to possibly regulate OPRL1, while hsa-miR-769-5p was found to possibly regulate NPP1. We believe that a multifactorial logistic regression model can be used to investigate the clinical significance of hsa-miR-630, hsa-miR-650, and hsa-miR-769-5p. Therefore, they were attempted to be included in this prediction model for further analysis. Ultimately, hsa-miR-769-5p was included in this prediction model. However, it has to be acknowledged that hsa-miR-769-5p was underweighted in this prediction model relative to hsa-miR-1258, hsa-miR-298, and hsa-miR-483-3p, suggesting that the potential mechanism of hsa-miR-769-5p regulation of NPP1 needs to be further validated.

In mammals, the natriuretic peptide is divided into three types, namely, A, B, and C. The three peptides are encoded by three separate genes, and *NPPA* is the coding gene for the ANP precursor [30, 31]. The *NPPA* gene is predominantly expressed in cardiac tissues, with low expression in other tissues (e.g., the lung, aorta, brain, adrenal gland, and uterus). To date, the underlying mechanisms of transcriptional regulation of *NPPA* in noncardiac tissues are not well understood [32]. *NPPA* mutations are associated with pulmonary infections; however, their detailed regulatory mechanisms are not known. In this study, the *NPPA* mRNA was found to be upregulated in BPD samples. hsa-miR-769-5p targets and regulates the *NPPA* mRNA and is a protective factor in BPD that promotes the degradation of NPPA mRNA and reduces the expression of ANP. The lungs are the main site for clearance of circulating ANP, which acts on T2 alveolar epithelial cells and inhibits the secretion of surface-active substances [33–38]. The lack of alveolar surface-active substances increases the surface tension of the alveoli and decreases compliance. Furthermore, overexpression of miR-769-5p inhibits the proliferation, migration, and invasion and promotes the apoptosis of keloid fibroblasts [39, 40]. miR-769-5p may inhibit fibrosis during BPD development, thus exerting a protective effect. In addition, miR1258 can inhibit the proliferation of many tumour cells in vivo, including non-small-cell lung cancer, liver cancer, and breast cancer [41–43]. To the best of our knowledge, in this study, miR1258 was found to be highly expressed in preterm infants with BPD for the first time and was identified as a risk factor for BPD. Furthermore, miR-483 may inhibit the proliferation and metastasis of glioma and colorectal cancer [44, 45]. It has been demonstrated that miR-483 targets insulin-like growth factor 1 (IGF1) and downregulates the expression of key proteins in the PI3K/AKT signalling pathway, thereby inhibiting myogenic cell proliferation and differentiation [46]. In the present study, miR483 was discovered to be highly expressed in the tissues of patients with BPD and may be involved in bronchial mucosal necrosis and poor repair after injury.

Bioinformatic analyses revealed that the neuropeptide-related gene *OPRL1* was upregulated in BPD samples. hsa-miR-650 and hsa-miR-630 had a targeting regulatory effect on *OPRL1* but were eventually not included in the prediction model owing to the insufficient number of relevant samples in the database. The nomogram prediction model established in this study requires to be verified in studies with large sample size for subsequent refinement of the results. Bioinformatic analyses in the present study were based on mRNA and miRNA data, and the corresponding gene and protein expression levels may not be consistent with the RNA expression levels. Protein content determination, and PCR assays, should be performed in future studies. It is worth noting that the mRNA dataset used is an umbilical cord tissue dataset and therefore the constructed exosomal miRNA-mRNA regulatory network has the potential to be biased and the reference to the relevant results needs to be used with caution. Overall, this study provides certain ideas for early clinical prediction of BPD by pooling multiple datasets.

## 5. Conclusions

A BPD prediction model based on hsa-miR-1258, hsa-miR-298, hsa-miR-483-3p, and hsa-miR-769-5p was constructed. Calibration curves demonstrated substantial agreement between the predicted and observed results of the model for BPD diagnosis. In addition, DCA revealed that the model had good clinical applicability. Therefore, the model can be used to predict the risk of BPD in newborns so that early diagnosis and prompt intervention can be implemented.

## Figures and Tables

**Figure 1:** Research design flow chart. The heat map represents the expression profiles of the final miRNAs used to construct diagnostic models in the training and validation groups. These miRNA signatures can distinguish between the samples of the BPD group and those of the control group (bottom right).

**Figure 2:** Volcano map of DEmiRNAs and heat map of RNA expression profiles in patients with BPD. (a) DEmiRNAs; (b) DEmRNAs. Purple dots represent upregulated RNAs. Blue dots represent downregulated RNAs. The five RNAs with the largest fold change are labelled in (a) and (b). (c) Heat map of differences in the expression of DEmiRNAs between the BPD and control groups; (d) heat map of differences in the expression of DEmRNAs between the BPD and control groups.

**Figure 3:** GO enrichment analysis of DEmRNAs and correlation heat map of DEmiRNAs in the ceRNA network. (a) The first five upregulated enriched GO pathways; (b) ten GO pathways that were significantly downregulated; (c) correlation analysis of DEmiRNAs in the ceRNA network.

**Figure 4:** The miRNA-mRNA ceRNA network. (a) Blue rectangles represent miRNAs, and red circles represent mRNAs. mRNA enrichment in the ceRNA network of upregulated (b) and downregulated (c) GO and KEGG pathways.

**Figure 5:** Expression of neuropeptides in the ceRNA network and their ability to classify BPD. (a) Sankey diagram demonstrating three miRNA-NP mRNA regulatory pairs in the ceRNA network; (b) differential expression of the neuropeptide-related genes *OPRL1* and *NPPA* between samples from the BPD and control groups; (c) the AUC values of the diagnostic classification ability of *OPRL1* and *NPPA* for BPD were shown; (d) gene set enrichment analysis (*GSEA*) of *OPRL1* indicates the KEGG CYTOKINE CYTOKINE RECEPTOR INTERACTION pathway and NABA ECM REGULATORS pathway are elevated. (e) GSEA of *NPPA* indicated the KEGG NEUROACTIVE LIGAND RECEPTOR INTERACTION pathway and the REACTOME ADORA2B MEDIATED ANTI INFLAMMATORY pathway.

**Figure 6:** Construction of SVM-RFE and lasso regression models and demonstration of classification performance. (a) A line graph between the number of incorporated variables and accuracy of the model during the training of the SVM-RFE model; the model had the highest accuracy when 11 variables were included; (b) the relationship between the choice of the penalty coefficient log(lambda) and retention variables in the lasso regression analysis; (c) using ten cross-validated lasso regression analyses, the relationship curves of binomial deviance and log(lambda) were drawn; 18 variables were selected for further analysis; (d) PCA demonstrating classification performance when the SVM-RFE model performs the best; (e) PCA demonstrating the classification performance of lasso logistic regression analysis.

**Figure 7:** Logistic regression analysis and the predictive power of the model. (a) Box plot depicting the differential expression analysis of four miRNAs between the BPD and control groups; (b) ROC curves demonstrating the classification performance of four miRNAs; (c) diagnostic prediction models were constructed using four miRNAs in the training set. Classification performance in the test and overall sets. (d) PCA of the prediction model constructed by those four miRNAs.

**Figure 8:** Construction and evaluation of a nomogram prediction model. (a) Nomogram for predicting the occurrence of BPD based on four miRNAs; (b) calibration curve showed the calibration of the prediction model between the predicted and observed values; (c) DCA curves demonstrating the range of safety and efficacy of the clinical prediction model.

**Table 1:** Chart of prediction factors.

Variable	*β*	Odds ratio (95% CI)	*P* value
(intercept)	-0.381	0.684 (0.207-2.041)	0.506
hsa-miR-1258	0.818	2.265 (1.438-3.862)	0.001
hsa-miR-298	-1.468	0.23 (0.085-0.53)	0.002
hsa-miR-483-3p	1.898	6.674 (2.832-20.003)	*P* < 0.001
hsa-miR-769-5p	-0.384	0.681 (0.284-1.488)	0.353

**Table 2:** Uni- and multilogistic regression analysis for predicting BPD.

Variables				
	Odds ratio (95% CI)	*P* value	Odds ratio (95% CI)	*P* value
hsa-miR-1258	1.658 (1.139-2.5)	0.011	2.207 (1.051-5.468)	0.051
hsa-miR-1293	2.097 (1.339-3.623)	0.003	1.535 (0.705-4.184)	0.329
hsa-miR-298	0.548 (0.33-0.87)	0.014	0.231 (0.034-1.126)	0.097
hsa-miR-302f	0.717 (0.514-0.991)	0.046	1.088 (0.603-2.039)	0.781
hsa-miR-3150b-3p	1.314 (1.066-1.662)	0.014	0.671 (0.326-1.198)	0.218
hsa-miR-325	1.558 (1.065-2.375)	0.029	1.782 (0.873-4.295)	0.135
hsa-miR-3605-5p	1.849 (1.191-3.082)	0.010	1.954 (0.715-7.046)	0.236
hsa-miR-483-3p	1.635 (1.096-2.65)	0.027	8.403 (1.846-82.04)	0.024
hsa-miR-514b-5p	2.141 (1.372-3.619)	0.002	1.57 (0.656-4.075)	0.321
hsa-miR-548n	0.738 (0.547-0.984)	0.041	0.732 (0.365-1.394)	0.345
hsa-miR-553	0.634 (0.426-0.906)	0.016	0.619 (0.304-1.095)	0.128
hsa-miR-650	0.739 (0.514-1.04)	0.088	1.26 (0.428-3.905)	0.668
hsa-miR-769-5p	0.715 (0.441-1.135)	0.156	0.312 (0.061-1.342)	0.13

## Data Availability

RNA profile data and clinical information for preterm infants with BPD were downloaded exclusively from the Gene Expression Omnibus (GEO) dataset (https://www.ncbi.nlm.nih.gov/geo/).

## Abbreviations

ANP: Atrial natriuretic peptide
AUC: Area under the curve
BPD: Bronchopulmonary dysplasia
DCA: Decision curve analysis
DEmiRNAs: Differentially expressed miRNAs
GEO: Gene Expression Omnibus
GO: Gene Ontology
GSEA: Gene Set Enrichment Analysis
KEGG: Kyoto Encyclopedia of Genes and Genomes
NICU: Neonatal intensive care unit
PCA: Principal component analysis
ROC: Receiver operating characteristic
SVM-RFE: Support vector machine-recursive feature elimination
VLBW: Very low birth weight.
